The article "When Words Hurt: Affective Word Use in Daily News Coverage Impacts Mental Health" was retracted in 2020. Reasons: errors in the data; errors in the methods; errors in the results or conclusions.

# When Words Hurt: Affective Word Use in Daily News Coverage Impacts Mental Health

**DOI:** 10.3389/fpsyg.2018.01333

**Published:** 2018-08-02

**Authors:** Jolie B. Wormwood, Madeleine Devlin, Yu-Ru Lin, Lisa Feldman Barrett, Karen S. Quigley

**Affiliations:** ^1^Department of Psychology, Northeastern University, Boston, MA, United States; ^2^School of Computing and Information, University of Pittsburgh, Pittsburgh, PA, United States; ^3^Department of Psychiatry, Massachusetts General Hospital, Athinoula A. Martinos Center for Biomedical Imaging, Charlestown, MA, United States; ^4^Edith Nourse Rogers Memorial (VA) Medical Center, Center for Healthcare Organization and Implementation Research, Bedford, MA, United States

**Keywords:** depression, mental health, startle reflex, news media, anxiety, physical symptoms

## Abstract

Media exposure influences mental health symptomology in response to salient aversive events, like terrorist attacks, but little has been done to explore the impact of news coverage that varies more subtly in affective content. Here, we utilized an existing data set in which participants self-reported physical symptoms, depressive symptoms, and anxiety symptoms, and completed a potentiated startle task assessing their physiological reactivity to aversive stimuli at three time points (waves) over a 9-month period. Using a computational linguistics approach, we then calculated an average ratio of words with positive vs. negative affective connotations for only articles from news sources to which each participant self-reported being exposed over the prior 2 weeks at each wave of data collection. As hypothesized, individuals exposed to news coverage with more negative affective tone over the prior 2 weeks reported significantly greater physical and depressive symptoms, and had significantly greater physiological reactivity to aversive stimuli.

Ample evidence has shown that the media influences people's mental and physical health, both intentionally, as in public health campaigns, and unintentionally (for a review, see Walsh-Childers and Brown, 2009). For instance, sensationalist reporting on suicides is associated with increased suicide rates (Niederkrotenthaler et al., 2012). Moreover, viewing distressing media footage following salient or evocative negative events, including incidents of mass violence, public health crises, and natural disasters, has been associated with increased posttraumatic stress symptoms (Bernstein et al., 2007; Holmes et al., 2007; Ben-Zur et al., 2012; Goodwin et al., 2013; Holman et al., 2014), psychological distress (Ben-Zur et al., 2012; Thompson et al., 2017), functional impairments (Thompson et al., 2017), higher incidence of mental and physical illnesses (Silver et al., 2013), and greater depressive symptom severity (Ahern et al., 2002). Indeed, media coverage of such salient or evocative negative events may impact mental health and well-being independently of any direct exposure to the event itself (e.g., Bernstein et al., 2007; Holmes et al., 2007; Silver et al., 2013). However, little has been done to examine the ways in which exposure to a broad range of news coverage from the mundane to the more affectively potent may impact mental and physical health among average adult community members in their everyday lives (although see McNaughton-Cassill, 2001).

Here, leveraging an existing three-wave dataset, we test the hypothesis that exposure to daily news content will be associated with changes in measures of mental health and well-being—and specifically, that exposure to news content that is more affectively negative in content or tone will be associated with poorer acute mental health symptoms, including increased physical symptoms, which have been shown to commonly co-occur with psychiatric conditions including mood and anxiety disorders (Kroenke et al., 1994, 2002), as well as increased depressive and anxiety symptoms. We posit that more regular or repeated exposure to modest daily stressors or negativity in the form of media content might have an additive effect resulting in acute increases in mental health symptoms among otherwise healthy adults.

Our hypothesis is also grounded in an emerging theoretical perspective concerning how the brain regulates energy balance both in the moment and in anticipation of future goals. Converging evidence from multiple disciplines suggests that the brain *anticipates* the body's needs and prepares to engage in optimized actions to satisfy those anticipated needs before they occur (Friston, 2010; Sterling, 2012; Barrett and Simmons, 2015; Sterling and Laughlin, 2015; Chanes and Barrett, 2016; Barrett, 2017a). The brain regions involved in tracking the body's immediate metabolic needs and likely future expenses—a balancing act known as allostasis (Sterling and Eyer, 1988; Sterling, 2012)—are also the brain regions typically associated with “affect” and “emotion” (sometimes referred to as “limbic” regions; Barrett and Simmons, 2015; Chanes and Barrett, 2016; Barrett, 2017a; Kleckner et al., 2017). These limbic brain regions are some of the most connected hubs in the entire brain, which scientists now consider the “backbone” of neural communication (see van den Heuvel and Sporns, 2011; Edlow et al., 2016; Barrett, 2017a). In the theory of constructed emotion (Barrett, 2017a,b), which guides this work, these limbic regions are hypothesized to issue the allostatic predictions about upcoming bodily needs which underlie all perception and action, modulating the activity of sensory, motor, and visceromotor neurons before incoming external sensory input reaches the brain (Barrett and Simmons, 2015; Chanes and Barrett, 2016; Barrett, 2017a,b; for a discussion of the tract-tracing studies that support this observation, see Barbas, 2015). Research has shown that when mediators of allostasis, such as neurotransmitters in the brain or hormones in the periphery, are overused due to excessive or repeated exposure to aversive stimuli, cumulative changes can lead to wear and tear on the brain and body called “allostatic load” (McEwen, 2003; Juster et al., 2010). Disruptions in allostasis and evidence of allostatic load have been implicated in emerging models of mood disorders, including depression (McEwen, 2003; Wilkinson and Goodyer, 2011; Barrett et al., 2016) and anxiety disorders such as post-traumatic stress disorder (PTSD; McEwen, 2003), as well as models of the impact of chronic stress on physical and mental health more generally (for a review, see Juster et al., 2010). Consistent with this theorizing, we posit that repeated exposure to negative or aversive news content on a regular basis may disrupt allostasis (i.e., the brain's ability to efficiently regulate the body in support of predicted energy needs), resulting in poorer mental and physical health.

In the present study, we test the hypothesis that individuals who were recently exposed to more affectively negative (less affectively positive) news content will exhibit poorer acute mental health symptoms. To test this, we analyzed an existing data set comprised of normal-functioning adults who were sampled three times (i.e., once during each of three waves of data collection) over approximately a 9-month period. At each wave of data collection, participants self-reported the written news sources to which they were exposed over the prior 2 weeks as well as how frequently they read content from each source. In addition, they self-reported their physical symptoms, depressive symptoms, and anxiety symptoms, and completed an affective modulation of startle task to assess their physiological reactivity to evocative, potentially aversive stimuli. We then utilized a computational linguistics approach to estimate the “affective tone” of the written news coverage to which each participant was recently exposed based on their self-reported news consumption. Specifically, we collected all of the actual written news content from the four most popular news sources reported by our sample over a 9-month period. We then quantified the proportion of affective words with positive and negative affective connotations in these articles (referred to as “affective tone”) and generated individualized measures for each participant at each wave of data collection by approximating the average affective tone of the daily news content read by a particular participant in the 2 weeks prior to each wave. We predicted that participants would self-report poorer mental health symptomology and have greater physiological reactivity when viewing evocative stimuli in the lab at times when their recent daily news exposure was more negative (less positive) in affective tone.

## Methods

### Participants

95 participants (36 males, 58 females, one undeclared) ages 17–61 (*M*_*age*_ = 28.29, *SD*_*age*_ = 10.58) from Northeastern University and the surrounding Boston community were recruited via advertisements on fliers posted around the city, on Craigslist.com, and in the Boston Metro newspaper for a study on threat perception and the Boston Marathon bombings. Potential participants completed the 8-item Patient Health Questionnaire (PHQ-8; Kroenke et al., 2009) and those without significant depressive symptomology (<10 on the PHQ-8) were eligible to participate. One additional participant was consented, but became syncopal during placement of the facial electromyography (fEMG) electrodes and withdrew from the experiment; no data was retained. Following this occurrence (after the first 30 participants had completed the first wave of data collection), potential participants were additionally screened for history of fainting in medical settings and all were offered a snack prior to beginning electrode placement at each session. Of the final sample, 57.9% identified as White, 13.7% identified as Black, 9.5% identified as Asian, 1.1% identified as Pacific Islander, 8.4% identified as more than one race, 5.3% identified as a race not listed, and 3.2% did not report their race. In addition, 12.6% identified as Hispanic, and 60.6% had some form of postsecondary education beyond high school. Thus, we were successful at recruiting a relatively diverse and representative sample from the Boston community.

These 95 participants were recruited to complete three waves of data collection surrounding the running of the annual Boston Marathon in April 2014, the first anniversary of the Boston Marathon bombings, with the first wave of data collection (Wave 1) between February 2, 2014, and March 12, 2014. 92 of these participants (96.8%) returned to complete the second wave of data collection (Wave 2) between March 31, 2014, and April 19, 2014, and 85 of these participants (89.5%) returned to complete the third wave of data collection (Wave 3) between September 10, 2014, and November 21, 2014 (with the exception of two of these 85 participants who instead completed it in June 2014 due to Fall conflicts). Participants received $30 for completing Wave 1, $40 for completing Wave 2, and $50 for completing Wave 3. Four participants were excluded from the sample prior to data analyses due to repeated failure to comply with experimental protocols across waves. Because analyses were completed using hierarchical linear modeling, which allows for missing data, participants who did not complete all three waves of data collection were retained in the sample for analyses, leaving a final sample of 91 participants.

Although sample size was not specifically determined *a priori* for the present analyses as we are leveraging an existing data set, multilevel analyses conducted using this sample size are considered appropriately powered to detect medium effect sizes. In multilevel designs, the upper-level (between-subject) sample size has more impact on the power than the lower-level (within-subject) sample size (i.e., number of participants affects power more than number of waves; Maas and Hox, 2005; Snijders, 2005), and simulation studies suggest that estimates of regression coefficients, standard errors, and variance components in multilevel models are generally accurate and unbiased with an upper-level sample size of approximately 100 for slopes of medium effect size (Maas and Hox, 2005).

### Procedure

At each wave of data collection, participants came to our laboratory at Northeastern University and completed a nearly identical experiment (with the exceptions noted in the task descriptions below). After providing informed consent (Wave 1 only), participants first completed a survey unrelated to the present investigation. They were then offered the option of taking a short break to have a snack (all except the first 30 participants of Wave 1) to minimize possible syncopal symptoms during fEMG electrode placement. Following this, fEMG electrodes were placed and participants completed the Affective Modulation of Startle Task (as described below). The fEMG electrodes were then removed and participants completed tasks unrelated to the present investigation. Finally, participants completed a set of questionnaires at the end of each experimental session which included measures of physical symptoms, depressive symptoms, and anxiety symptoms. Participants were debriefed in-person at the end of their third experimental session or were sent a debriefing statement via e-mail if they did not complete Wave 3.

### Tasks and measures

#### Affective modulation of startle task

We assessed participants' physiological reactivity to potentially aversive stimuli by measuring the startle blink reflex in a potentiated acoustic startle paradigm. The startle blink reflex is potentiated by aversive states or contexts and reduced by affectively pleasant states or contexts (for a review, see Grillon and Baas, 2003). In our task, participants listened to a series of 24 white noise bursts (~95 dB, 50 ms, instantaneous rise time) over binaural headphones while electromyographic (EMG) activity was recorded over the *orbicularis oculi* muscle region under the left eye. These white noise bursts, called startle probes, occurred while the participants were viewing images on the computer. They viewed 28 images in a random order: 14 neutral images from the International Affective Picture Set (IAPS; Lang et al., 2008) and 14 images taken from media coverage of a recent local terrorist attack, the Boston Marathon bombings (e.g., from the *Boston Globe*, the *Boston Metro*, or the *New York Times*). Images of the Boston Marathon bombings were specifically selected to be ambiguous in terms of the level of threat they might engender in viewers. For example, one image showed a first responder carrying an injured woman to safety, which could be conceptualized as uplifting (if attending to the first responder) or as threatening/aversive (if attending to the injured woman). All images were displayed for 6 s with a jittered inter-image interval of 10–16 s during which a white fixation cross was displayed in the middle of a black screen. To reduce the predictability of startle probe presentations, two images of each type were presented without a startle probe, and startle probes were presented at quasi-random intervals following image onset (3–5 s after image onset) on the remaining 24 trials. After Wave 1, half of the images of each type were replaced with novel images of the same type, as past research suggested this may improve the reliability of measures of the affective modulation of startle (Larson et al., 2000). However, we found no differences in the reliability of reactivity measures calculated using novel vs. familiar images following Wave 2, and thus we retained the same images in this task from Waves 2 to 3.

The primary dependent variable was *startle modulation*, or the difference in the amplitude of the reflexive startle blink response on trials where the startle probe was presented during evocative (i.e., terrorism-related) images vs. during presentation of neutral images. Because our terrorism-related images were specifically selected to be ambiguous in terms of how aversive or positive they might be to viewers, we anticipated that we would find both positive and negative values for startle modulation (i.e, not all participants would exhibit more pronounced startle responses to the terrorism-related images than to the neutral images). Here, positive values of startle potentiation indicate a more pronounced startle response while viewing the terrorism-related images than the neutral images, indicating the terrorism-related images were perceived as more aversive or threatening. Conversely, negative values indicate a less pronounced startle response while viewing the terrorism-related images than the neutral images, indicating the terrorism-related images were perceived more positively (e.g., as uplifting images of first responders).

#### fEMG acquisition and processing

To assess the amplitude of the reflexive startle blink response, activity of the orbicularis oculi muscle was assessed using facial electromyography (fEMG) techniques. Two reusable Ag/AgCl electrodes from Mindware Technologies LTD (Gahanna, OH) were filled with a conductive electrolyte gel (Signal Gel; BioMedical Instruments; Warren, MI) and placed over the orbicularis oculi muscle region under the participant's left eye with a reference electrode in the middle of the forehead. To ensure proper signal conductivity, each site was cleaned with alcohol before electrode placement and the area for the reference electrode placement was also exfoliated using a semi-abrasive lotion. Muscle activity was sampled at 1,000 Hz using BioLab v. 3.0.13 (Mindware Technologies LTD; Gahanna, OH), using BioLab's default EMG filter (gain of 5,000, low cutoff of 20 Hz, and high cutoff of 200 Hz). Mindware's EMG scoring software (v3.1.0I) was used to process the fEMG signal whereby the rectified raw fEMG signal was smoothed with a rolling filter (*f*_*c*_ = 16 Hz). The mean amplitude (in microvolts) of the processed signal in the 40 ms before each startle probe was taken as a baseline measure of muscle activity for that trial. To calculate the startle blink amplitude for each trial, this baseline value was subtracted from the peak amplitude of the processed signal in the epoch from 0 to 200 ms following the presentation of the startle probe. All raw data was subject to visual inspection by trained scorers who identified individual trials for exclusion from analyses, including trials with blink activity during the baseline period, trials with multiple blinks following the presentation of the startle probe, trials with blinks within 0–40 ms after presentation of the startle probe (which is too early to be the reflexive startle blink), or trials with unusual signal characteristics (e.g., movement artifact or signal noise caused by improper electrode placement or skin preparation). Participants who did not have at least 12 scoreable trials were removed from analyses involving this task. Useable startle data was obtained from 80 participants at Wave 1 (84.2%), 86 participants at Wave 2 (93.5%), and 79 participants at Wave 3 (92.9%). For these remaining participants, trial-by-trial data exclusions as a result of the aforementioned criteria accounted for 2.2% of all data at Wave 1, 2.6% of Wave 2 data, and 3.7% of Wave 3 data. As in other potentiated startle tasks (see, for example, Lang et al., 1990), we assessed the degree of potentiation of the startle response when viewing potentially aversive (i.e., terrorism-related) images relative to more neutral images. For each participant, the mean amplitude of the startle blink reflex across all trials during neutral images was subtracted from the mean amplitude of the startle blink reflex across all trials during terrorism-related images to create the measure of *startle modulation*.

### Questionnaires

#### Demographic information

At Wave 1 only, participants completed a questionnaire that assessed their age, gender, ethnicity, race, and education level.

#### Physical symptoms

At each wave, participants completed the Patient Health Questionnaire-15 (PHQ-15), which measures non-specific physical symptoms that commonly co-occur with psychiatric conditions (Kroenke et al., 1994, 2002) and also are commonly elevated after major life stressors like a combat deployment or other potentially traumatic event (Clauw et al., 2003; van den Berg et al., 2005). At each wave of data collection, participants rated the severity of 15 physical symptoms (e.g., back pain, stomach pain) over the past 4 weeks on a scale from 0 to 2, where 0 is “Not Bothered at All,” 1 is “Bothered a Little,” and 2 is “Bothered a Lot.” Responses were summed to yield a total physical symptom severity score for each wave.

#### Depressive symptoms

At each wave, participants completed the 8-item Personal Health Questionnaire (PHQ-8; Kroenke et al., 2009). The PHQ-8 is used to detect and measure the severity of depressive symptoms primarily in research studies. Participants reported how often they were bothered by a list of symptoms over the past 2 weeks (e.g., “little interest or pleasure in doing things” and “feeling down, depressed, or hopeless”). Responses were given on a scale from 0, “Not at All,” to 3, “Nearly Every Day.” Responses to individual items were summed to yield a single score indicating the severity of depressive symptoms at each wave.

#### Anxiety symptoms

At each wave, participants completed the 21-item Beck Anxiety Inventory (BAI; Beck and Steer, 1993). The BAI consists of 21 symptoms (e.g., heart pounding/racing, nervous, indigestion) that are rated on a 4-point severity scale referring to the experience of symptoms over the past month (from 0, “Not at All,” to 3, “Severely Bothered Me”). Scores for the 21 items were summed to yield a single state anxiety symptom score for each wave.

#### Neuroticism

At Wave 1 only, participants also completed the shorter version of the Revised NEO Personality Inventory (NEO-PI-R) called the NEO Five Factor Inventory (NEO-FFI; Costa and MacCrae, 1992). The NEO-FFI contains 60 items in total, 12 items to assess each of five factor domains: neuroticism, extraversion, openness to experience, agreeableness, and conscientiousness. Participants rated the degree to which they agreed with statements about themselves (e.g., “I am not a worrier”) on five-point scales (from 1, “Very Slightly or Not at All”, to 5, “Extremely”). After reverse-scoring applicable items, the 12 items for each factor were averaged to give a single score for each factor. For the present analyses, we focus on the neuroticism subscale of the NEO-FFI given its relationship to the frequency and intensity of negative affective experience (see, for example, Costa and McCrae, 1980) and to both mental and physical symptoms (e.g., Bienvenu and Stein, 2003; Deary et al., 2007; Klein et al., 2011).

#### Media usage questionnaire

At each wave of data collection, participants were asked to list all sources that they used over the past 2 weeks to obtain news, including any newspapers (online and print), television shows, social media sites, and radio programs. For each source they listed, participants also rated the frequency with which they used that news source over the past 2 weeks on a five-point scale, where 1 = “Only once”; 2 = “A few times”; 3 = “Most days”; 4 = “Every day”; and 5 = “Multiple times per day”.

### Analysis

#### Deriving a time- and usage-dependent measure of affective tone in news coverage

We first identified the four most frequent news outlets participants reported using on the Media Usage Questionnaire at Waves 1 and 2: *The Metro (MT), The New York Times (NY), The Boston Globe (BG)*, and *The Boston Herald (BH)*. Other outlets, such as *USA Today* and the *Wall Street Journal*, were each reported by fewer than 10 respondents. Therefore, our data collection focused on the news content published by the four most frequently reported outlets. We used Google News, a news aggregator website, to retrieve news articles published by these four outlets on a daily basis. We first collected the URLs of the news articles from Google News, and retrieved and parsed the news content using the Java HTML parser, jsoup (jsoup.org). The data were drawn from a period of about 2 weeks before each participant participated in the study at each wave until a few days after the end of each wave. Because media data collection occurred concurrently with in-lab data collection, we gathered content from all sources for some additional days at each wave in order to ensure we had appropriate coverage of all relevant media data for all participants for all waves. Data collected on these additional days were never utilized in the data analyses. Table S1 in the Supplemental Material shows the durations of each wave, the duration of media data collection for each wave, and a summary of the media data collected. In total, we collected over 38.5 K news articles covering the three waves of the study.

To measure the affective tone of this media coverage, we first identified the number of words with positive and negative affective connotations in each article. Identification of affective words and the classification of affective words as negative or positive was determined using the psycholinguistic lexicon Linguistic Inquiry and Word Count (LIWC; Pennebaker et al., 2015). We then calculated a sentiment ratio (*SR*): the ratio of the number of positive words (*P*) to the total number of positive (*P*) and negative words (*N*) for each article [*SR* = *P*/(*P* + *N*)]. We did not use the simpler ratio *P/N* because this ratio could be arbitrarily large, which can result in misleading analyses/models. We then took the average of this sentiment ratio, *SR*, from all news articles published on each day *t* from each outlet, where this daily average for each outlet is given by: *SR*_*O*_(*t*). To address data sparseness, we then employed a rolling average for this variable, creating a smoothed variable, ${\tilde{SR}}_{O}\left(t\right)$, such that: ${\tilde{SR}}_{O}\left(t\right)=\frac{1}{\delta }\underset{t\;-\;\delta <t^{{\;}^{\prime }}<t}{\sum }{\tilde{SR}}_{O}\left(t^{\prime }\right)$, where δ is chosen to be 7 days in this study and *t*′ is a running variable indicating the range of the smoothing (from *t* – δ to *t*, for each *t*). Next, the smoothed variable, ${\tilde{SR}}_{O}\left(t\right)$, was re-scaled from −1 to 1, where −1 indicates that, over the time period δ (i.e., 7 days), all affective words were negative, 1 indicates that all affective words were positive, and 0 indicates an equivalent number of positive and negative affective words. Plots of ${\tilde{SR}}_{O}\left(t\right)$, for each outlet, for each wave can be found in Figure S1 in the Supplemental Material.

Finally, to capture “recent exposure” to affective news coverage *for each participant at each wave*, we: (1) took the average of ${\tilde{SR}}_{O}\left(t\right)$, for each outlet, over only the 14 days prior to each participant's in-lab session, and then (2) took a weighted average across the four outlets, such that the values for each outlet at each wave were weighted by the participant's self-reported usage of each outlet at that wave (as reported in the Media Usage Questionnaire at each wave). Thus, for each wave (*w*), each participant (*i*) had a single variable (*X*_*wi*_) that reflected the affective tone (i.e., the proportion of positive and negative affective word usage) in recent news coverage (i.e., in only articles published within the 2 weeks prior to their in-lab session within wave (*w*)) from only the news sources that the participant personally reported having used over those past 2 weeks. We refer to this individualized variable as the *affective tone of recent news coverage exposure*. Higher values indicate increases in the proportion of positive affective words and decreases in the proportion of negative affective words, while lower values indicate decreases in the proportion of positive affective words and increases in the proportion of negative affective words in articles from news sources participants reported being exposed to in the 14 days prior to their in-lab session for each wave of data collection.

#### Modeling impact of affective tone on mental health

To examine whether changes in the affective tone of the news coverage to which each participant was recently exposed predicts corresponding changes in that individual's mental health symptoms, we analyzed our data using hierarchical linear modeling (HLM; Raudenbush and Bryk, 2002; Raudenbush et al., 2011). This approach has advantages over traditional methods of analyzing repeated-measures data (e.g., repeated-measures ANOVA), including simultaneous estimation of within-subject and between-subject variance, more efficient estimation of effects, and lower Type-1 error rates (Kenny et al., 2003). For our primary analyses, all models were of the general form:

(1) $$\begin{array}{r} Y_{wi}=\pi_{0i}+\pi_{1i}\left(X_{wi}\right)+e_{wi} \end{array}$$

where

(2) $$\begin{array}{r} \pi_{0i}=B_{00}+r_{0i} \end{array}$$

and

(3) $$\begin{array}{r} \pi_{1i}=B_{10}+r_{1i} \end{array}$$

where *Y*_*wi*_ refers to the outcome variable (i.e., physical symptoms, depressive symptoms, anxiety symptoms, or startle modulation) collected at the in-lab session for wave (*w*) nested within participant (*i*); *X*_*wi*_ refers to the affective tone of news coverage to which participant (*i*) reported being exposed in the 2 weeks prior to their in-lab session within wave (*w*); *e*_*wi*_ refers to the wave-level error, *B*_00_ and *B*_10_ refer, respectively, to population-value estimates for the intercept and slope linking the affective tone of recent news coverage exposure to the outcome variable; and *r*_0*i*_ and *r*_1*i*_ refer, respectively, to the participant-level variability in the intercept and slope values (i.e., across-participant variability).

These analyses were completed using the HLM 7 software package for hierarchical linear and nonlinear modeling from Scientific Software International, Inc. (Raudenbush et al., 2011), utilizing a continuous sampling model with a restricted maximum likelihood method of estimation for model parameters and parameter estimates calculated with robust standard errors. Following the recommendation of Enders and Tofighi (2007), throughout the analyses, all Level-1 variables (i.e., wave-level variables, like mental health symptom reporting or affective tone of recent news coverage) were centered around each participant's own across-wave mean, and all Level-2 variables (i.e., participant-level variables like age, gender, and neuroticism) were centered around the sample mean (i.e., “grand mean centered”).

## Results

As shown in Table 1, the HLM analyses revealed that when participants were exposed to news coverage with more positive (less negative) affective tone over the prior 2 weeks, they reported significantly fewer physical symptoms [*B*_10_ = −4.80, *SE* = 1.86; *t*_(90)_ = 2.58, *p* = 0.012; see Figure 1A] and significantly fewer depressive symptoms [*B*_10_ = −4.06, *SE* = 1.69; *t*_(90)_ = 22.40, *p* = 0.018; see Figure 1B] but not significantly fewer anxiety symptoms [*B*_10_ = −2.25, *SE* = 2.60, *t*_(90)_ = 0.87, *p* = 0.389; see Figure 1C]. Participants exposed to recent news coverage with more positive (less negative) affective tone also exhibited significantly lower startle modulation values [*B*_10_ = −6.82, *SE* = 3.03; *t*_(90)_ = 2.25, *p* = 0.027; see Figure 1D], suggesting less physiological reactivity to potentially aversive (i.e., terrorism-related) images relative to neutral images. Estimates of variance components for each model are given in Table S2 in the Supplemental Material.

**Table 1:** Changes in affective tone of recent news coverage exposure predict mental health symptoms and startle modulation.

**Outcome**	***B***	***SE***	***t*-ratio**	***df***	***p***	**Cohen's *d***
**PHYSICAL SYMPTOMS**						
*B_00_*	3.57	0.27	13.29	90	<0.001^*^	2.80
*B_10_*	−4.80	1.86	2.58	90	0.012^*^	0.54
**DEPRESSIVE SYMPTOMS**						
*B_00_*	2.71	0.24	11.43	90	<0.001^*^	2.41
*B_10_*	−4.06	1.69	2.40	90	0.018^*^	0.51
**ANXIETY SYMPTOMS**						
*B_00_*	3.80	0.35	10.83	90	<0.001^*^	2.28
*B_10_*	−2.25	2.60	0.87	90	0.389	0.18
**STARTLE MODULATION**						
*B_00_*	−0.41	0.59	0.69	90	0.489	0.15
*B_10_*	−6.82	3.03	2.25	90	0.027^*^	0.47

*Model coefficients are unstandardized. B_00_ and B_10_ refer, respectively, to population-value estimates for the intercept and slope linking the affective tone of recent news coverage exposure to each outcome variable*.

* *p < 0.05*.

**Figure 1:** Simple slopes representation of models predicting changes in mental health symptoms and startle potentiation from changes in the affective tone of recent news coverage exposure. Models predicting physical symptoms **(A)**, depressive symptoms **(B)**, anxiety symptoms **(C)**, and startle modulation **(D)** from affective tone of recent news coverage exposure. Values for affective tone indicate the proportion of affective words that were positive and negative in the recent news coverage (i.e., over the previous 2 weeks) to which participants reported being exposed. Higher values for affective tone indicate increases in the proportion of positive affective words and decreases in the proportion of negative affective words, while lower values for affective tone indicate decreases in the proportion of positive affective words and increases in the proportion of negative affective words. Model slopes are represented by a black line, with ±1 standard error of the slope and intercept for each model shown as a gray shaded area. SD stands for standard deviation.

Critically, exposure to recent news coverage with a more positive (or less negative) affective tone remained a significant within-person predictor of physical symptoms, depressive symptoms, and startle modulation when controlling for individual differences in age, gender, and neuroticism (see Table 2).

**Table 2:** Changes in affective tone of recent news coverage exposure predicts mental health symptoms and startle modulation controlling for age, gender, and neuroticism.

**Outcome**	***B***	***SE***	***t*-ratio**	***df***	***p***	**Cohen's *d***
**PHYSICAL SYMPTOMS**						
*B_00_* (Intercept)	3.57	0.27	13.29	90	<0.001^*^	2.80
*B_10_* (Affective tone)	−4.87	1.93	2.52	87	0.014^*^	0.54
*B_11_* (Age)	0.08	0.20	0.38	87	0.705	0.08
*B_12_* (Gender)	1.50	3.34	0.45	87	0.655	0.10
*B_13_* (Neuroticism)	1.98	3.31	0.60	87	0.552	0.13
**DEPRESSIVE SYMPTOMS**						
*B_00_* (Intercept)	2.71	0.24	11.43	90	<0.001^*^	2.41
*B_10_* (Affective tone)	−4.13	1.71	2.42	87	0.018^*^	0.52
*B_11_* (Age)	0.17	0.19	0.87	87	0.390	0.19
*B_12_* (Gender)	2.07	2.90	0.72	87	0.477	0.15
*B_13_* (Neuroticism)	1.42	3.19	0.45	87	0.657	0.10
**ANXIETY SYMPTOMS**						
*B_00_* (Intercept)	3.89	0.35	10.84	90	<0.001^*^	2.29
*B_10_* (Affective tone)	−2.72	2.69	1.01	87	0.314	0.22
*B_11_* (Age)	0.11	0.31	0.37	87	0.711	0.08
*B_12_* (Gender)	5.86	4.41	1.33	87	0.187	0.29
*B_13_* (Neuroticism)	−1.50	4.24	0.35	87	0.724	0.08
**STARTLE MODULATION**						
*B_00_* (Intercept)	−0.41	0.59	0.69	90	0.491	0.15
*B_10_* (Affective tone)	−7.14	3.03	2.36	87	0.020^*^	0.65
*B_11_* (Age)	0.37	0.26	1.41	87	0.161	0.30
*B_12_* (Gender)	0.57	6.44	0.09	87	0.930	0.02
*B_13_* (Neuroticism)	6.30	4.94	1.28	87	0.205	0.27

*All models were of the general form: Ŷ_wi_ = π_0i_ + π_1i_(X_wi_) + e_wi_, where π_0i_ = B_00_ + r_0i_ and π_1i_ = B_10_ + B_11_(Age_i_) + B_12_(Gender_i_) + B_13_(Neuroticism_i_) + r_1i_; Y_wi_ refers to the outcome variable (i.e., physical symptoms, depressive symptoms, anxiety symptoms, or startle modulation) collected at the in-lab session for wave (w) nested within participant (i); X_wi_ refers to the affective tone of news coverage to which participant i reported being exposed in the two weeks prior to their in-lab session within wave (w); e_wi_ refers to the wave-level error, B_00_ and B_10_ refer, respectively, to population-value estimates for the intercept and slope linking the affective tone of recent news coverage exposure to the outcome variable controlling for all other variables (i.e., age, gender, neuroticism); B_11_, B_12_, and B_13_ refer, respectively, to population-value estimates for the change in the slope of B_10_ as a function of age, gender (dummy-coded), and neuroticism; r_0i_ and r_1i_ refer, respectively, to the participant-level variability in the intercept and slope values (i.e., across-participant variability). Model coefficients are unstandardized*.

* *p < 0.05*.

Descriptive statistics and zero-order correlations between variables are available in Tables S3 and S4 in the Supplemental Material.

## Discussion

Exposure to news media is psychologically impactful. Individuals in our study reported fewer physical and depressive symptoms and were less physiologically reactive to potentially aversive stimuli when they had been exposed to news coverage characterized by a less negative (more positive) affective tone over the prior 2 weeks, even when controlling for individual differences in age, gender, and neuroticism. This also means that those exposed to news coverage characterized by a more negative (less positive) affective tone over the prior 2 weeks reported more physical and depressive symptoms, and were more physiologically reactive to potentially aversive stimuli. Thus, over and above the *content* of what was reported (such as suicides or incidents of mass violence), fluctuations in the affective connotation of daily news coverage predicted changes in well-being.

The finding that affective tone co-varied with startle modulation is particularly compelling, as it suggests that physiological reactivity to evocative images may change as a function of exposure to varying affective word usage in recent news media. In particular, because we selected evocative images for our startle task that were ambiguous in terms of the amount of threat they might engender in viewers, our findings suggest that changes in the affective tone of recent news coverage exposure may be associated with changes in the *interpretation* of affectively ambiguous, potentially threatening images. For instance, it is possible that individuals who read news content containing a higher proportion of affectively negative words experienced the terrorism-related images as more threatening (e.g., by focusing on the destruction or injuries of victims in the photos), while individuals who read news content containing a higher proportion of affectively positive words experienced the terrorism-related images as more uplifting (e.g., by focusing on the heroics of first responders in the photos). However, the present work is correlational in nature and cannot speak to causality. Future research should experimentally test whether repeated exposure to news content with a more negative affective tone can bias one's perception of and physiological reactivity to evocative images.

The news, whether pleasant or unpleasant, has the ability to expand a person's “affective niche”—it has the ability to make events outside of one's immediate surroundings personally-relevant, granting them the capacity to impact that person's well-being. One's affective niche includes everything in their physical and psychological environment that is relevant to that person's allostasis (Barrett, 2017a; although see Colombetti and Krueger, 2015, for an alternative definition of this term). Exposure to news coverage expands our affective niche to encompass events from around the globe—it makes us cheerful, compassionate, or even angered by people and events on the other side of the world. A larger affective niche may at times benefit allostasis via social regulation by helping us feel connected to people and places who are remote during times of pleasant news. However, this expansion also carries the cost of potential allostatic disruption, particularly when news content is unpleasant or even threatening. Just as changes to the physical environment can be disruptive and impose new selection pressures on an organism (i.e., negative niche construction; Laland et al., 2000), so too can changes in the affective environment. If disruptions to allostasis persist, they can result in poorer mental and physical health, with both short- and long-term consequences for an individual (Barrett and Simmons, 2015; Barrett et al., 2016).

Although our findings are consistent with the idea that news exposure can expand one's affective niche and disrupt allostasis, it is important to note that the present study is correlational and cannot test causal explanations. An alternative possibility, for instance, is that individuals with greater current physical and depressive symptoms actively seek out news content that is less affectively positive or more affectively negative. Indeed, the present sample may be biased such that it over-represents individuals willing to seek-out and engage with news content that is more affectively negative: the current study leveraged an existing sample specifically recruited for a study related to a local terrorist attack (i.e., the Boston Marathon bombings), and participants were told they would be viewing images of the attack during the study. Future experimental research should directly test this alternative explanation by examining news content selection among a representative sample of individuals with varying levels of physical and depressive symptom severity.

Future research should also extend the present findings to alternative measures of both media exposure and mental health and well-being. For example, future research could include more objective behavioral indicators of mental health and well-being (e.g., physical activity, voice tone, reaction time), as well as objective physical health outcomes related to persistently disrupted allostasis (e.g., increases in cardiovascular dysregulation and dysfunction; Blascovich and Katkin, 1993; Williams and Medlock, 2017). In addition, in the present study, we designed our media exposure variable to balance concerns about objectivity and specificity in assessing media exposure. Our operationalization focused on specific outlets that our participants reported reading recently and weighted the contribution of each news outlet based on each participant's self-reported usage of that news outlet. We did not, however, assess participants' perceptions of the affective tone of the articles or their potentially biased memory for which specific content they read over the past 2 weeks. It would be interesting for future research to compare the present method to one that more heavily prioritizes specificity or granularity in measuring media exposure. For instance, because our approach does not ask participants about which specific articles they actually read from each news source over the prior 14 days, there is no guarantee that the average affective tone of a given news outlet reflects the average affective tone of the specific articles each person actually read from that outlet. In this way, our findings may actually underestimate the strength of the relationship between mental health symptoms and the affective tone of recent news coverage exposure, and future research should examine this possibility.

Contrary to predictions, we did not find a significant relationship between the affective tone of recent news coverage exposure and anxiety symptoms in the present study, though the relationship was in the predicted direction. One possibility for this null result is that anxiety symptoms (in comparison to physical or depressive symptoms) are related to exposure to more specific emotion content beyond affective valence. For example, perhaps recent exposure to threatening or fear-inducing content (e.g., a shooting or a public health crisis) might increase the frequency of anxiety symptoms although exposure to more general negative content in the present study did not. This would be consistent with previous findings that effects of general negativity can be distinguished from those of threat (Kveraga et al., 2015; Boshyan et al., 2018). Future research should examine the impact of more specific emotion content in news media, beyond affective valence, to reveal novel relationships with mental health and well-being and with anxiety symptoms in particular.

Another possibility is that anxiety symptoms are related to exposure that is more affectively negative than observed in the present study. That is, news content in the present study included, on average, more words with positive than negative affective connotations (see Figure S1 in the Supplemental Material). As the relative proportion of affectively negative words increased, we saw associated increases in physical symptoms, depressive symptoms, and physiological reactivity, but in general there were still more positive than negative affective words used by each news outlet as a whole for each day. It is possible that anxiety symptoms are only associated with affective tone once the overall content is more negative on the whole. Future experimental work should examine how the observed relationships between affective tone and mental health are moderated by the average affective tone of the news content to which participants have recently been exposed.

Finally, future research should also expand to investigate the psychological and physical health impacts of affective tone in additional types of news media. The present study focused on exposure to written, verbal affective content in newspapers, and so it is unclear whether our findings extend to news media formats that are potentially more immersive, such as radio, television, or social media sites. While we would hypothesize that exposure to affectively negative words would impact mental and physical health symptoms across these different modalities, it seems likely that news media sources with additional channels for conveying affective meaning beyond verbal content (e.g., vocal prosody, bodily movement, and evocative imagery) might produce even stronger relationships between news exposure and mental health symptoms. Moreover, platforms like Facebook and Twitter have become ubiquitous parts of daily life for a large portion of the population—people can now receive breaking news content continuously throughout the day right in the palm of their hand. Yet, much remains unknown about social media use and its impact on the construction of our affective niches and allostasis. For example, social media use is associated with reporting greater depressive symptomology (Lin et al., 2016) and lower levels of happiness (Brooks, 2015), but can also facilitate feelings of connection and social support (Lin and Margolin, 2014; Neubaum et al., 2014). Future research should examine whether the affective tone of the media content to which individuals are being exposed on social media determines when and for whom social media use is beneficial vs. detrimental to well-being.

## Conclusion

It is the media's job to report on events in the world that people might find upsetting. But our findings suggest that exposure to news content using vivid, negatively toned language for attention-grabbing purposes is associated with detrimental changes in readers' mental health symptom severity that may persist for weeks. Importantly, however, our findings suggest that not only is exposure to more negative (less positive) news coverage associated with evidence of disrupted allostasis, but that exposure to more positive (less negative) news coverage is associated with evidence of more efficient allostasis (i.e., with beneficial changes in mental health symptomology and physiological reactivity). These findings are consistent with the possibility that news coverage with more positive affective tone may buffer individuals against the distress caused by negative news content (e.g., related to crime, disease, natural disasters, terrorism) that must be conveyed.

## Ethics statement

This study was carried out in accordance with the recommendations for the basic ethical principals of respect for persons, beneficence, and justice as set forth in the Belmont Report. These principles are codified in 45 Code of Federal Regulations Part 46, subparts A–D—Protection of Human Subjects. The protocol was approved by Northeastern University's Institutional Review Board. All subjects gave written informed consent in accordance with the Declaration of Helsinki.

## Author contributions

JW, YRL, LFB, and KQ contributed to study design and funding acquisition. JW collected and processed the behavioral and physiological data and YRL collected, analyzed, and processed the media signaling data. JW conducted data analyses with input from all other authors. MD and JW drafted the manuscript and all authors helped edit the manuscript.

### Conflict of interest statement

The authors declare that the research was conducted in the absence of any commercial or financial relationships that could be construed as a potential conflict of interest.
